The article "A Regulatory Mechanism Involving TBP-1/Tat-Binding Protein 1 and Akt/PKB in the Control of Cell Proliferation" was retracted in 2019. Reasons: manipulated images; duplicated data; unreliable results or conclusions; concerns about the data.

# A Regulatory Mechanism Involving TBP-1/Tat-Binding Protein 1 and Akt/PKB in the Control of Cell Proliferation

**DOI:** 10.1371/journal.pone.0022800

**Published:** 2011-10-04

**Authors:** Maria Sepe, Luisa Festa, Fabio Tolino, Luca Bellucci, Luca Sisto, Daniela Alfano, Pia Ragno, Viola Calabrò, Vittorio de Franciscis, Girolama La Mantia, Alessandra Pollice

**Affiliations:** 1 Dipartimento di Biologia Strutturale e Funzionale, Università di Napoli “Federico II”, Naples, Italy; 2 Istituto per l'Endocrinologia e l'Oncologia Sperimentale del Consiglio Nazionale delle Ricerche (CNR) “G. Salvatore”, Naples, Italy; 3 Dipartimento di Chimica, Università degli Studi di Salerno, Salerno, Italy; Florida International University, United States of America

## Abstract

TBP-1 /Tat-Binding Protein 1 (also named Rpt-5, S6a or PSMC3) is a multifunctional protein, originally identified as a regulator of HIV-1-Tat mediated transcription. It is an AAA-ATPase component of the 19S regulative subunit of the proteasome and, as other members of this protein family, fulfils different cellular functions including proteolysis and transcriptional regulation. We and others reported that over expression of TBP-1 diminishes cell proliferation in different cellular contexts with mechanisms yet to be defined. Accordingly, we demonstrated that TBP-1 binds to and stabilizes the p14ARF oncosuppressor increasing its anti-oncogenic functions. However, TBP-1 restrains cell proliferation also in the absence of ARF, raising the question of what are the molecular pathways involved. Herein we demonstrate that stable knock-down of TBP-1 in human immortalized fibroblasts increases cell proliferation, migration and resistance to apoptosis induced by serum deprivation. We observe that TBP-1 silencing causes activation of the Akt/PKB kinase and that in turn TBP-1, itself, is a downstream target of Akt/PKB. Moreover, MDM2, a known Akt target, plays a major role in this regulation. Altogether, our data suggest the existence of a negative feedback loop involving Akt/PKB that might act as a sensor to modulate TBP-1 levels in proliferating cells.

## Introduction

TBP1/Tat-Binding Protein 1 (also named Rpt-5, S6a or PSMC3) is a member of a large highly conserved gene family of ATPases (ATPAses Associated to a variety of cellular Activities) whose key feature is a highly conserved module of 230 aa consisting of an ATPase and a DNA/RNA helicase motif. This protein family fulfils a large diversity of cellular functions including cell cycle regulation, gene expression, vesicle mediated transport, peroxisome assembly and proteasome function [1]. Indeed, as other members of the family, TBP-1 is associated with the 19S regulatory subunit of the proteasome, the chief site of protein destruction in eukaryotic cells [2]. The last 10 years have highlighted the essential role of proteolysis in governing cell physiology. Protein breakdown is required not only for removal of abnormal or aged proteins, but also to control most biological pathways through the regulated degradation of key cellular factors. Moreover, abnormal proteasome expression levels have been described in many tumor cells and proteasome plasma levels appear elevated in neoplastic patients, underlying the involvement of the proteasome in cancer development [3], [4]. Consistent with the role in protein destruction, TBP-1 has been shown to bind the tumour suppressor VHL (Von-Hippel-Landau) gene product [5] contributing to its E3-ubiquitin ligase function towards the Hif1-a factor, thus acting as a *bona fide* tumor suppressor.

The article "A Regulatory Mechanism Involving TBP-1/Tat-Binding Protein 1 and Akt/PKB in the Control of Cell Proliferation" was retracted in 2019. Reasons: manipulated images; duplicated data; unreliable results or conclusions; concerns about the data.

On the other hand, 19S protein components (TBP-1 among them) behave as multifaceted proteins, being implicated in different cellular events that do not require proteolysis like transcriptional initiation and elongation, [6], [7], [8] Nucleotide Excision Repair [9] and regulation of mitosis [10].

We and others have reported that TBP-1 may function as a negative regulator of cell proliferation: inhibition of the oncogenic phenotype of *erb-B* transformed cells was accompanied by an increase of TBP-1 intracellular levels and, accordingly, its overexpression in *erb-B* transformed cells strongly inhibited tumour formation in athymic mice [11]; furthermore, TBP-1 overexpression in different cellular contexts diminished cell proliferation [11], [12]. Our reported results [12], [13] showing that TBP-1 enhances the levels of the p14ARF oncosuppressor well fit with TBP-1 proposed antioncogenic role [11]. On the other hand, the observation that TBP-1 overexpression can inhibit cell proliferation also in ARF minus contexts [11], [12] suggests an ARF-independent role of TBP-1, raising the question of what molecular pathways may be involved.

In this paper, we address the role of TBP-1 in the control of cell proliferation. To this aim we used, as model, a primary human fibroblast cell line immortalized by h-TERT (human telomerase) expression where p14ARF levels are undetectable and in which we have silenced the expression of TBP-1. Our results show that cellular levels of TBP-1 are critical in the control of cell proliferation pointing to a functional relationship between TBP-1 and the Akt/PKB serine-threonine kinase, one of the major transducers of growth signals mediating proliferative and pro-survival effects.

## Results

### TBP-1 depletion determines an increase in the growth properties

We decided to first study the effects of long term silencing of TBP-1 in an immortalized human fibroblast cell line (T11hT). To this purpose, by retrovirus infection, we generated stable T11hT-derived cell clones that constitutively express a *sh-*RNA specifically designed to silence TBP-1 expression (see Materials and Methods). As shown in Figure 1A, TBP-1 is efficiently silenced in six stable clones analyzed, with an extent of silencing ranging from 80% to 48%. To exclude that reduced expression of TBP-1 may have altered proteasome assembly and function [14], we analyzed intracellular levels of proteasome subunits other than TBP-1 in three of the silenced clones (T1, T10E and T10C). In all cases we observed that the levels of expression of three different proteasome subunits (Rpt-6, Rpt-1 of the 19S subunit and C8 of the 20S subunit) do not change significantly as compared to parental T11hT (Figure 1B). Furthermore, we didn't observe any variation of the *in vitro* proteasome activity of cell extracts obtained from TBP-1-silenced clones and parental cells on two different peptide substrates (data not shown).

The article "A Regulatory Mechanism Involving TBP-1/Tat-Binding Protein 1 and Akt/PKB in the Control of Cell Proliferation" was retracted in 2019. Reasons: manipulated images; duplicated data; unreliable results or conclusions; concerns about the data.

**Figure 1:** Characterization of TBP-1 silenced clones. **A, B:** Cells stably transfected with TBP1 *sh*-RNA plasmid or control cells (wt T11hT, Human Primary Fibroblasts Immortalized by hTERT) were cultured in DMEM+10%FBS for 24 hrs. Levels of TBP-1 expression was evaluated by Western Blot with anti-TBP-1 on whole protein lysates. **B**: As control, protein levels of other proteasome components (two 19S-ATPases, Rpt-1 and Rpt-6, and a 20S component, C8) was evaluated in the clones T1, T10C and T10E. Bands intensity was evaluated by ImageQuant analysis on at least two different expositions to assure the linearity of each acquisition, each normalised for the respective actin values. Asterisk, fold value is expressed relative to the reference point (i.e. TBP-1 levels in T11hT cells), arbitrarily set to 1. Representative of at least four independent experiments.

We then measured the growth rate of the T1 and T10C clones as compared to that of the T11hT cells. Figure 2A shows that both the TBP-1 silenced clones analysed proliferate at higher rate respect to the parental T11hT cell line. In particular, the T1 clone, expressing very low TBP-1 levels (see Figure 1), grows at a rate that is roughly twice that of the parental cell line. Moreover, serum deprivation doesn't appreciably alter the growth rate of the silenced clones (Figure 2B). To exclude any clonal secondary effect due to the selection process, we also generated, by stable transfection, T11hT cell pools either containing the *sh*-TBP-1 vector or the empty vector. As it is shown in Figure 2C and D, TBP-1 silenced cells, although in a less pronounced way respect to single clones, display the same growth profile, both in presence and absence of serum.

The article "A Regulatory Mechanism Involving TBP-1/Tat-Binding Protein 1 and Akt/PKB in the Control of Cell Proliferation" was retracted in 2019. Reasons: manipulated images; duplicated data; unreliable results or conclusions; concerns about the data.

**Figure 2:** TBP-1 knockdown determines an increase in the growth properties. **A, B:** Cells from the T1, T10C and control cells (wt T11hT) were cultured in DMEM either in the presence (**A**) or in absence (**B**) of 10% FBS. Cells were collected at the time points indicated and counted in a Burker chamber. The values are the mean ± SE of three experiments performed in triplicate. **C, D**: wt T11hT cells, cells from control cell pool or from the *sh*-TBP-1 cell pool were cultured in DMEM either in the presence (**C**) or in absence (**D**) of 10% FBS. Cells were collected at the time points indicated and counted in a Burker chamber. The values are the mean ± SE of three experiments performed in triplicate. **E, F:** Cells from the T1 clone were transfected by electroporation with empty vector (indicated just as T1) or TBP-1 expression plasmid (indicated as T1+TBP-1); cells were then cultured either in the presence (**E**) or in absence (**F**) of 10%FBS and collected at the time points indicated (being T_0_ the time at 24 hours after transfection). Cells from each time point have been counted in a Burker chamber. Values are mean ± SE of two experiments performed in triplicate and are indicated as values relative to the reference point (T_0_). **E, F lower panels**: TBP-1 expression and Akt activation have been evaluated by Western Blot with anti-TBP-1, anti-Phospho-Akt Ser473, anti-Akt and anti-actin, as loading control, on whole protein lysates of cells collected at each time point, as indicated.

The enhanced growth rate in TBP-1 silenced cells seems to be dependent on TBP-1 silencing. In fact, transient expression of TBP-1 in the faster proliferating T1 clone dramatically reduces its proliferation rate, both in presence (Figure 2E) and absence (Figure 2F) of serum; however, after 48 hrs, when the expression of exogenous TBP-1 was greatly reduced (see Figure 2E and F, lower panels), cells start to proliferate faster suggesting that slow proliferating TBP-overexpressing cells were selected against.

Consistently with the ability of TBP-1 silenced clones to actively proliferate even in the absence of serum, the cell viability of the T1 clone, measured after 6 hrs of serum withdrawal, remains high. In particular, T11hT cell viability was reduced from 60% to 10% (depending on cell density), while that of the T1 clone is reduced only up to 60% at the lowest cell density (Figure 3A and B). We thus investigated whether TBP-1 silencing may increase cell resistance to serum withdrawal-induced apoptosis. As shown in Figure 3C and D, the T1 clone behaves more resistant to serum-deprivation, respect to the parental cells, as assessed by the very faint amounts of both Caspase-3 and PARP-1 cleavage. Accordingly, flow cytometry analysis indicates that serum starvation only slightly affects the percentage of T1 cells in S phase (8% reduction), while more drastically reduces that of the parental cell line (55% reduction) (Figure 3E). Furthermore, the increase of the sub-G1 population (of around 1.8 fold for the T1 clone and 3,14 fold for the parental cell line) is consistent with PARP-1 and Capase-3 cleavage data (Figure 3E and see 3C and D).

The article "A Regulatory Mechanism Involving TBP-1/Tat-Binding Protein 1 and Akt/PKB in the Control of Cell Proliferation" was retracted in 2019. Reasons: manipulated images; duplicated data; unreliable results or conclusions; concerns about the data.

**Figure 3:** TBP-1 knockdown reduces sensitivity to serum starvation. **A, B:** Cells from the T1 clone and control cells (wt T11hT) were plated at different cell densities as indicated, either in the presence or absence of 10% FBS. After six hrs from plating, cell viability was measured by MTS assay. In the histograms, cell viability is expressed as relative to controls, arbitrarily set to 100 (%). The values are the mean ± SE of three experiments performed in quintuplicate. **C, D:** 1.8×10^5^ cells/35 mm plates from the T1 clone and control cells (wt T11hT) were grown for 24 hrs, in the presence or absence of 10% FBS. Apoptosis was checked by detection of Caspase-3 (**C**) and PARP-1 (**D**) cleavage in Western Blot. Detection with anti-actin was included for control of equal loading. Bands Intensity was measured by ImageQuant analysis on at least two different expositions to assure the linearity of each acquisition. Representative of at least four independent experiments. **E:** T11hT and T1 cells were counted and seeded at 2×10^5^cells/35 mm plate. At 24 hrs cells were collected and treated for analysis of cellular DNA content by flow cytometry. Percentages of cells in the SubG1, G0–G1, S and G2–M phases were quantified with Summit 4.1 software. Representative of three different experiments. The numerical ratios reported on the right highlight the different behaviour of T1 cells when grown in absence or presence of serum. Table 1 provides the mean values (and standard deviations in parentheses) relative to this analysis.

**Table 1:** Mean values (and standard deviations in parentheses) relative to the flow cytometry analysis described in Figure 3.

	T11hT+serum	T11hT−serum	T1+serum	T1−serum
**Sub-G1**	**12,69** (+/−2,35)	**39,79** (+/−5,02)	**13,02** (+/−1,8)	**29,05** (+/−3,12)
**S**	**14,87** (+/−1,2)	**6,44** (+/−0,9)	**13,94** (+/−1,75)	**14,13** (+/−2,49)

Next, we analyzed the invading capability of the T1 clone respect to control cells by a chemoinvasion assay in which cells were plated on Matrigel coated filters and allowed to migrate. As shown in Figure 4A, as compared to parental cells, T1 cells possess a moderate but significant higher ability to migrate through Matrigel. Interestingly, similar results are also obtained when cells were allowed to migrate toward a generic chemoattractant as EGF (Epidermal Growth Factor) (Figure 4B). To further prove that the difference in invasion ability could be ascribed to the reduction of TBP-1 protein levels and not to any clonal secondary effects, making use of a specific *si*RNA, we transiently silenced TBP-1 in parental T11hT cells. Consistently, transient silencing of TBP1 is even more effective than stable silencing in T1 cells in inducing a high per cent of migrating cells (Figure 4C). Thus, the difference in Matrigel invasion was likely due to an increased invading capability of TBP1 silenced cells, as also suggested by the fact that we don't observe any difference both in the expression and activation status of the EGF receptor (not shown).

The article "A Regulatory Mechanism Involving TBP-1/Tat-Binding Protein 1 and Akt/PKB in the Control of Cell Proliferation" was retracted in 2019. Reasons: manipulated images; duplicated data; unreliable results or conclusions; concerns about the data.

**Figure 4:** Silencing of TBP-1 determines an increase of the invading capability. **A:** Cells from the T1 clone or control cells (wt T11hT) were plated in Boyden chambers and allowed to migrate on filters coated with Matrigel. The values are the mean ± SE of three experiments performed in triplicate. (*) p = 0.046 as determined by the Student's t test. **B:** Cells from the T1 clone or control cells (wt T11hT) were plated in Boyden chambers and allowed to migrate toward EGF on Matrigel filters. 100% values represent cell migration in the absence of chemoattractants. The values are the mean ± SE of three experiments performed in triplicate. (*) p = 0.027 as determined by the Student's t test. **C:** Cells transiently transfected with TBP1 *si*-RNA or with the control si-RNA (*si*-Luc) were plated in Boyden chambers and allowed to migrate toward EGF on filters coated with Matrigel. 100% values represent cell migration in the absence of chemoattractants. The values are the mean±SE of three experiments performed in triplicate. (*) p = 0.016 as determined by the Student's t test.

Taken together these data show that TBP-1 sensitizes cells to apoptosis induced by serum withdrawal and interferes with cell growth and migration.

### TBP-1 inhibits Akt/PKB activation

The observation that TBP-1 depletion allows cells to grow in a serum-independent manner, prompted us to ask whether TBP-1 expression levels may control, in some way, the activity of the Akt/PKB serine-threonine kinase, one of the major transducers of growth signals, critical for cell proliferation and apoptosis. We thus evaluated the levels of phospho-Akt in our TBP-1 depleted clones, under actively growth conditions (i.e. in the presence of serum). As shown in Figure 5A, pAkt/PKB levels are inversely correlated to the extent of silencing of TBP-1, being the lowest in the parental T11hT and the highest in the T1 clone. Consistently, we observed an increase in the extent of phosphorylation of GSK3β, a well characterized Akt/PKB direct target. TBP-1 reduction appears to specifically affect Akt activation but not that of other important transducers of growth signals, like ERK_1/2_. Furthermore, in agreement with the observed higher proliferation rate of the clones, we observed a reduction of phospho-cyclin D1 protein levels (data not shown). Both in parental cells and in TBP-1 silenced clones, Akt activation appears to be dependent on the upstream phosphatidylinositol 3-kinase activity (PI3K) as evidenced by Wortmannin and LY294002 treatment that block PI3K activity (Figure 5B).

The article "A Regulatory Mechanism Involving TBP-1/Tat-Binding Protein 1 and Akt/PKB in the Control of Cell Proliferation" was retracted in 2019. Reasons: manipulated images; duplicated data; unreliable results or conclusions; concerns about the data.

**Figure 5:** TBP-1 knockdown determines activation of the Akt/PKB kinase. **A:** Cells from the T1, T10C and control cells (wt T11hT) were cultured in DMEM+10%FBS for 24 hrs. Activation of Akt/PKB was revealed by Western Blot with anti-Phospho-Akt Ser473 antibody. As control, extracts were also probed with anti-Akt, anti-Phospho-GSK-3β/pSer219, anti-pERK_1/2_, anti-ERK_1/2_ and anti-actin antibodies. Bands Intensity was measured by ImageQuant analysis on at least two different expositions to assure the linearity of each acquisition, each normalised for the respective actin values. Asterisk, fold value is expressed relative to the reference point, arbitrarily set to 1. Representative of at least four independent experiments. **B:** Cells from the T1 clone or control cells (wt T11hT) were plated at the cell density of 2.5×10^5^ in DMEM+10%FBS in six wells. After 24 hrs, either DMSO (/) or with Wortmannin or LY294002, where indicated, were added to the cells at the concentrations indicated and left for either 1 hour (with Wortmannin) or 15′(with LY294002). Extracts were then probed in Western Blot with antibodies against Akt, Phospho-Akt Ser473 and actin. **C, D:** T11hT cells (**C**) or U2OS cells (**D**) were transfected with an *si*RNA directed against TBP-1 or Luciferase. Extracts were probed with antibodies against Phospho-Akt Ser473, Akt and actin. **E:** Cells from the T1 clone were transfected with empty vector (first lane) or increasing amounts of TBP-1 expression plasmid. Activation of Akt/PKB was evaluated by Western Blot on whole protein lysates probed with anti-Phospho-Akt Ser473 and, as control, with anti-Akt and anti-actin. **F:** U2OS cells were transfected with empty vector (lanes 1–4) or TBP-1 expression plasmid (lanes 5, 6). After 24 hrs cells were starved for 4 hrs and treated with 10 ng/ml insulin for 10′ where indicated. Activation of Akt/PKB was evaluated by Western Blot on whole protein lysates probed with anti-Phospho-Akt Ser473. Extracts were also probed with anti-Akt, anti-actin and anti-Xpress (to reveal transfected TBP-1).

The article "A Regulatory Mechanism Involving TBP-1/Tat-Binding Protein 1 and Akt/PKB in the Control of Cell Proliferation" was retracted in 2019. Reasons: manipulated images; duplicated data; unreliable results or conclusions; concerns about the data.

Importantly, we could reproduce, in T11hT cells, the same effect after transient reduction of TBP-1 levels by *si*RNA: silencing of TBP-1 was accompanied by a concomitant increase in the steady-state level of pAkt, suggesting the existence of a causal relationship between TBP-1 intracellular levels and Akt activation (Figure 5C). This effect was not cell-specific since we could reproduce it in the U2OS osteosarcoma-derived cells (Figure 5D).

Further, we set up a rescue experiment in which we re-established high TBP-1 levels in the T1 clone by transient overexpression. In these conditions we observed a strong reduction of pAkt levels (Figure 5E and see also Figure 2E, F). Consistently, insulin-mediated activation of Akt in a different cellular context (U2OS cells) is counteracted by TBP-1 overexpression (Figure 5F). Altogether these data suggest that TBP-1 levels modulate the extent of Akt/PKB activation.

### TBP-1 is a downstream target of Akt activation

The new insights into the role of TBP-1 in the control of cell growth prompted us to investigate whether TBP-1 protein levels are sensitive to acute growth factors stimulation. We thus stimulated either T11hT or U2OS osteosarcoma cells by insulin treatment for the indicated time periods and analyzed protein lysates by Western Blots with anti-TBP-1 antibodies. Figure 6A clearly shows that insulin treatment results in a rapid, transient drop of TBP-1 intracellular levels; indeed, TBP-1 levels are reduced of around two times in 5 min and remain low up to 40 minutes with a kinetic that mirrors that of the activation of Akt/PKB (Figure 6A, left panel). On the other hand, other proteasome subunits (Rpt-6 and C8) protein levels remain almost stable or, at least, slightly increased, following insulin treatment (Figure 6A). To test the effects of inhibition of the PI3K/Akt pathway on TBP-1 protein levels, U2OS cells or T11hT cells were treated for the indicated time periods with PI3K inhibitors and protein lysates analyzed by Western Blots. As shown in Figure 6B, inhibition of the PI3K/Akt pathway determines a slight though reproducible increase in TBP-1 endogenous levels, suggesting that they are either directly or indirectly regulated by PI3K activity. Again, in these conditions, other proteasome subunits (Rpt-6 and C8) protein levels remain stable (Figure 6B, left panel). To further confirm these observations, we transiently transfected increasing amounts of a constitutively active mutant of the Akt kinase (CA-Akt) in U2OS cells. Overexpression of CA-Akt was accompanied by a reduction of endogenous TBP-1 levels, while other proteasome subunits protein levels remain unchanged (Figure 6C). Taken together, these data strongly indicate that TBP-1 protein levels are modulated by the Akt/PKB activity.

The article "A Regulatory Mechanism Involving TBP-1/Tat-Binding Protein 1 and Akt/PKB in the Control of Cell Proliferation" was retracted in 2019. Reasons: manipulated images; duplicated data; unreliable results or conclusions; concerns about the data.

**Figure 6:** TBP-1 is a downstream target of Akt activation. **A:** U2OS cells or T11hT cells were starved for 4 hrs and then treated with 10 ng/ml insulin for the times indicated. Activation of Akt/PKB was evaluated by Western Blot on whole protein lysates probed with anti-Phospho-Akt Ser473 and anti-Akt. Levels of endogenous TBP-1 and of two proteasome components (C8 and Rpt-6) were analyzed where indicated. TBP-1 bands intensity was measured by ImageQuant analysis on two different expositions to assure the linearity of each acquisition, each normalised for the respective actin values. Asterisk, fold value is expressed relative to the reference point, (i.e. TBP-1 levels in starved cells) arbitrarily set to 1. Representative of three independent experiments. **B:** U2OS cells or T11hT cells were treated, 24 hrs after plating, either with DMSO (/) or with 200 nM Wortmannin or 50 mM LY294002 for the times indicated. Cells were then lysed and Western Blot analysis was performed by using specific antibodies against Phospho-Akt Ser473, anti-Akt, anti-TBP-1, anti-C8 and anti-Rpt-6. TBP-1 bands intensity was calculated as in A. Representative of three independent experiments. **C:** U2OS cells were transfected with empty vector (lane 1) or increasing amounts of the constitutive active mutant of the Akt kinase (CA-Akt). After 24 hrs cells were lysed and whole cell lysates probed with anti-Phospho-Akt Ser473, anti-Akt, anti-TBP-1, anti-Rpt-1, anti-Rpt-6, and anti-phospho-GSK3b. **D:** U2OS cells were transfected with a *si*RNA directed against MDM2 or Luciferase, as control, at the final concentration of 10 nM. After 24 hrs, cells were starved for 4 hrs and then treated with 10 ng/ml insulin for the times indicated. Cells were then lysed and Western Blot analysis was performed by using specific antibodies against Phospho-Akt Ser473, TBP-1, MDM2, Akt, and actin. **E:** U2OS cells were transfected with a *si*RNA directed against MDM2 or Luciferase, as control. After 48 hrs, either DMSO (/) or 200 nM Wortmannin was added to the cells and left for the times indicated. Cells were then lysed and Western Blot analysis was performed by using specific antibodies against Phospho-Akt Ser473, TBP-1, MDM2, Akt and actin.

On the other hand, by immunoprecipitation experiments we were unable to observe any physical interaction between TBP-1 and Akt/PKB (data not shown), suggesting that TBP-1 levels are indirectly modulated by Akt activation. We thus wondered which could be the mediator of Akt/PKB action on TBP-1.

The article "A Regulatory Mechanism Involving TBP-1/Tat-Binding Protein 1 and Akt/PKB in the Control of Cell Proliferation" was retracted in 2019. Reasons: manipulated images; duplicated data; unreliable results or conclusions; concerns about the data.

Among the known Akt/PKB effector is the MDM2 protein that, following phosphorylation by Akt/PKB, increases its activity [15], [16], [17]. We thus determined whether MDM2 mediates the functional relationship between TBP-1 and Akt/PKB. In order to obtain Akt activation, we treated with insulin U2OS cells that were previously either treated with a MDM2 specific *si*RNA or, as control, with a luciferase *si*RNA (Figure 6D). Interestingly, MDM2 silencing prevented the reduction of TBP-1 intracellular levels following treatment with insulin, although has no effects on TBP-1 basal levels. Consistently, the increase in TBP-1 levels following treatment with PI3K inhibitors, is prevented in cells in which MDM2 is silenced (Figure 6E), suggesting that, indeed, silencing of MDM2 renders Akt activation/inactivation ineffective on TBP-1 levels. These data strongly implicate MDM2 to be needed, even not sufficient, for TBP-1 regulation by Akt/PKB. Involvement of MDM2 is supported by co-immunoprecipitation experiments in U2OS cells. As shown in Figure 7A and 7B we found TBP-1 in complex both with endogenous and with transfected MDM2. Furthermore, we observed that overexpression of MDM2 causes a decrease of TBP-1 intracellular levels (Figure 7A and B, see *input*). We confirmed this observation transfecting U2OS cells with fixed concentration of pcDNA-TBP-1 and increasing amounts of the MDM2 expression plasmid (Figure 7C). Since the observed effect occurs both on the endogenous and on the exogenous protein, it is likely that MDM2 acts on TBP-1 at the post-transcriptional level. Moreover, treatment of U2OS cells with the proteasome inhibitor MG132 counteracts the MDM2 effect on TBP-1, indicating the proteasome as the final effector of the MDM2 action on TBP-1 (Figure 7D).

**Figure 7:** TBP-1 is a downstream target of MDM2 activation. **A:** U2OS cells were either transfected (lanes +) or untransfected (lanes −) with the MDM2 expression plasmid. 24 hrs after transfection cell extract was prepared and subjected either to immunoprecipitation with anti-TBP-1 antibody where indicated or, with anti-GFP antibody as negative control. Cell extracts were also incubated with protein A-agarose as control, where indicated. Immunoprecipitated extracts were analyzed by Western Blot with anti-MDM2 or anti-TBP-1 antibody. Aliquots of cell extracts were analyzed by Western Blot before immunoprecipitation (*input*). **B:** U2OS cells were either transfected (lanes +) or untransfected (lanes −) with the MDM2 expression plasmid. 24 hrs after transfection cell extract was prepared and subjected either to immunoprecipitation with anti-MDM2 antibody where indicated or, with anti-Flag antibody as negative control. Cell extracts were also incubated with protein A-agarose as control, where indicated. Immunoprecipitated extracts were analyzed by Western Blot with anti-MDM2 or anti-TBP-1 antibody. Aliquots of cell extracts were analyzed by Western Blot before immunoprecpitation (*input*). **C:** U2OS cells were transfected with TBP-1 expression plasmid and increasing amounts of MDM2 expression plasmid. After 24 hrs, cells were lysed and whole cell extracts probed with anti-TBP-1, anti-MDM2, and anti-actin, for loading control. **D:** U2OS cells were transfected with TBP-1 expression plasmid and increasing amounts of MDM2 expression plasmid. After 24 hrs cells were treated either with DMSO (first four lanes) or with 10 µM MG132 where indicated. Cell extracts were analyzed by Western Blot with anti-Xpress (to reveal transfected TBP-1), anti-MDM2, and anti-actin, for control. **E:** U2OS cells were transfected with TBP-1 expression plasmid and increasing amounts of either MDM2_wt_, MDM2_S166A_ or MDM2_S166A/S186A_ expression plasmids. After 24 hrs cells were lysed and whole cell extracts were analyzed by Western Blot with anti-Xpress (to reveal transfected TBP-1), anti-MDM2, and anti-actin, for control. **F:** U2OS cells were transfected with TBP-1 expression plasmid and increasing amounts of either MDM2_wt_, MDM2_1–441_ or MDM2_Δ150–230_ expression plasmids. After 24 hrs cells were lysed and whole cell lysates analyzed by Western Blot with anti-Xpress (to reveal transfected TBP-1), anti-MDM2, and anti-actin, for control.

The article "A Regulatory Mechanism Involving TBP-1/Tat-Binding Protein 1 and Akt/PKB in the Control of Cell Proliferation" was retracted in 2019. Reasons: manipulated images; duplicated data; unreliable results or conclusions; concerns about the data.

We thus asked if mutations in MDM2 that render it less responsive to Akt/PKB stimulation [15], [16], [17], [18] reduces, as well, its ability to downregulate TBP-1 levels. The MDM2_S166A_ and MDM2_S166A/186A_ mutants appear almost unable to mediate TBP-1 degradation (Figure 7E), indicating that only a functionally Akt-responsive MDM2 molecule, could regulate TBP-1 levels. Accordingly, a MDM2 deletion mutant that lacks all the Akt target sites in MDM2 (MDM2_Δ150–230_) [19] appear unable to act on TBP-1 levels (Figure 7F). Interestingly, a MDM2 mutant, lacking the ring finger domain (MDM2_1–441_), is still able to act on TBP-1 (Figure 7F), indicating that MDM2 is not acting on TBP-1 levels through its ubiquitination activity.

These data provide clear evidence that TBP-1 is a downstream target of the Akt/PKB-MDM2 axis, even though the molecular mechanisms through which MDM2 acts on TBP-1 remain to be elucidated.

The article "A Regulatory Mechanism Involving TBP-1/Tat-Binding Protein 1 and Akt/PKB in the Control of Cell Proliferation" was retracted in 2019. Reasons: manipulated images; duplicated data; unreliable results or conclusions; concerns about the data.

## Discussion

Herein we report data showing that reduction of TBP-1 intracellular levels affects cell proliferation, invading capabilities and resistance to apoptosis of human fibroblasts immortalized by h-TERT expression. Interestingly, unlike the parental cells, proliferation of TBP-1 silenced clones appears to be serum-independent. Our data indicate that TBP-1 modulates the extent of activation of the Akt/PKB kinase, a critical effector of intracellular signaling. In fact, we demonstrate that reduction of TBP-1 intracellular levels causes the activation of the Akt signaling pathway. It has to be underlined that this can be directly ascribed to TBP-1 depletion rather than to clonal secondary effects as it also occurs after transient silencing of TBP-1 and irrespective of the cell type. Remarkably, transient expression of TBP-1 in one of the silenced clones restores phospho-Akt basal levels and drastically reduces the proliferation rate. Furthermore, TBP-1 overexpression in other cellular systems prevents Akt/PKB activation thus confirming that TBP-1 can act upstream of Akt.

Activation of the Akt/PKB pathway plays a central role in tumorigenesis. Indeed, Akt is overexpressed in many different tumour cell types, with a burgeoning list of substrates implicated in oncogenesis [20]. In principle, the increase of Akt/PKB activity could account for all the changes induced by TBP-1 silencing (i.e. proliferation, cell viability, escape from apoptosis, migration capabilities) [21], [22], [23], [24]. On the other hand, the acquisition of a transformed phenotype is a quite complex stepwise accumulation of genetic changes [25], [26]. In this context, it seems plausible to predict that, by acting on Akt/PKB, down-modulation of TBP-1 intracellular levels might contribute to the acquisition of a transformed phenotype thus cooperating with other genetic lesions. Since TBP-1 silenced clones are normal fibroblasts that only bear h-TERT overexpression to guarantee immortalization, an intriguing possibility to explore is the introduction of “key” cellular lesions to cause cell transformation in these clones.

The mechanism by which TBP-1 prevents Akt/PKB activation remains an open question. Even though, like the other AAA-ATPases of the 19S base of the proteasome, TBP-1 is supposed to act by conferring specificity to the proteasome [27], [28] various observations suggest that TBP-1 may act, as well, in a proteasome independent manner [6], [7], [8], [12], [13], [29]. Indeed, the proteasome seems very unlikely involved in the modulation of the Akt/PKB activity by TBP-1. In fact, an increase in the proliferation rate is frequently associated to an increase of proteasome levels needed to guarantee high metabolic activity. Here we show that TBP-1 silenced clones don't display a significant alteration in proteasome composition and activity. Furthermore, unlike other proteasome components (C8 and Rpt-6), TBP-1 responds to acute insulin stimulation with a decrease of its intracellular levels. In a different context, other proteasome subunits respond to growth factor stimulation with an increase of intracellular levels [30].

The article "A Regulatory Mechanism Involving TBP-1/Tat-Binding Protein 1 and Akt/PKB in the Control of Cell Proliferation" was retracted in 2019. Reasons: manipulated images; duplicated data; unreliable results or conclusions; concerns about the data.

It has to be underlined that we have already observed that TBP-1 stabilizes p14ARF [12], [13] avoiding ARF entrance into the proteasome. We retain that TBP-1 could play a role in ARF folding, rendering it a poor substrate for degradation by the 20S as well as by the 20S/11S proteasome [31], [32]. The existence of a similar mechanism that permits to TBP-1 to increase the intracellular levels of proteins that regulate Akt/PKB activity is the subject of further studies.

Furthermore, our results reveal the existence of a reciprocal regulatory loop where Akt/PKB activation leads to TBP-1 reduction and, in turn, TBP-1 overexpression prevents Akt/PKB activation. In this scenario, the Akt/PKB kinase thus might act as a sensor that modulates TBP-1 levels in actively duplicating cells. On the other hand, based on the fact that the PI3K/Akt signaling effect on TBP-1 is prevented in cells in which MDM2 is silenced, we propose, as mediator of the PI3K/Akt signaling on TBP-1, the MDM2 protein, one of the main direct targets of Akt/PKB activation [15], [16], [17], [18]. Actually, MDM2 can bind to TBP-1 and its overexpression causes a reduction of TBP-1 intracellular levels. Strikingly, the MDM2_S166A/S186A_ mutant and the MDM2_Δ150–230_, lacking Akt responsive sites, are unable to act on TBP-1 protein levels, likely placing TBP-1 downstream of the Akt/PKB-MDM2 axis.

Even though the specific mechanism for MDM2-dependent depression of TBP-1 levels remains to be understood, it has to be noted that MDM2 has multifaceted roles in protein degradation. In fact, aside its well-described role as E3-ubiquitin ligase, under appropriate stimuli, MDM2 can shuttle p63 to the cytoplasm mediating its interaction with proteins specifically involved in its turnover [33]. Moreover, MDM2 has been shown to mediate proteasome-dependent but ubiquitin-independent degradation of p21^Waf1/Cip1^ [19] and of Retinoblastoma Protein [34] through direct binding with the C8 subunit of the 20S proteasome. On the other hand, it has very recently been reported that MDM2 interacts with components of the 19S proteasome in a ubiquitylation independent manner [35] claiming a wider view of its mechanism of action.

Interestingly, the MDM2_Δ150–230_ mutant was described to be unable to shuttle between the nucleus and the cytoplasm, displaying a predominant cytoplasmic localization [19]. This could imply that the MDM2 action on TBP-1 levels requires its nuclear localization that, indeed is described to occur following phosphorylation by Akt [15], [18].

The article "A Regulatory Mechanism Involving TBP-1/Tat-Binding Protein 1 and Akt/PKB in the Control of Cell Proliferation" was retracted in 2019. Reasons: manipulated images; duplicated data; unreliable results or conclusions; concerns about the data.

Moreover, the fact that the MDM2_1–441_ deletion mutant, that lacks the ring finger domain, is still able to act on TBP-1 (Figure 7F), indicates that MDM2 is not acting on TBP-1 levels through its ubiquitination activity, supporting the possibility that it rather acts as a molecular cargo and should plausibly act in concert with other pAkt effector molecule(s) needed to direct TBP-1 for degradation.

Altogether our observations provide further insights on the proposed antiproliferative role of TBP-1 [11], [12], [13], indicating the involvement of the Akt/PKB kinase. Indeed, we could speculate that, under standard growing conditions, TBP-1 contributes to balance Akt/PKB up-regulation; whilst, under growth factor acute stimulation, activation of the Akt/PKB signaling pathway lowers TBP-1 levels and initiate a feedback loop. Further, it's interesting to underline that the human oncosuppressor p14ARF that is stabilized by TBP-1 overexpression [12], [13] is itself able to antagonize the activity of Akt/PKB [36] with yet unknown mechanism. On the other hand, other reports [37] underline an *in vivo* requirement of ARF for full activation of PTEN, one of the major negative regulators of Akt activity.

In conclusion, our data well support a role for TBP-1 in the attenuation of Akt/PKB activity and place this protein with a key role in the control of cell proliferation. Even though, further studies are necessary to understand the potential cross-talks linking TBP-1 action on p14ARF and on Akt/PKB regulation.

## Materials and Methods

### Cell cultures, viral infection, transfections

T11hT (human primary fibroblasts immortalized by constitutive expression of the telomerase catalytic subunit h-TERT) human cell line was kindly provided by dr. Eric Gilson. T1, T10C and T10E (TBP-1 silenced clones) derived by retroviral infection of T11hT: briefly, 3×10^6^ HEK 293-LinX packaging cells (kindly provided by Prof. Nicola Zambrano) were transfected with ARREST-IN (Open Biosystems, Huntsville, AL, USA) with pSUPERIOR.shTBP-1. 24 hrs after transfection, virus containing supernatant was filtrated through 0,45 µm cellulose acetate syringe filter, supplemented with 5 µg/ml polybrene, and used to infect recipient T11hT cells, previously plated at 50% confluence. Twenty-four hours following infection, 1 mg/ml G418 was applied to select stably infected cells. After three weeks, 23 individual single G418 resistant clones were picked up and expanded. Six neomycin resistant colonies from 5 different plates, were screened by Western Blot with anti-TBP-1.

The article "A Regulatory Mechanism Involving TBP-1/Tat-Binding Protein 1 and Akt/PKB in the Control of Cell Proliferation" was retracted in 2019. Reasons: manipulated images; duplicated data; unreliable results or conclusions; concerns about the data.

Both T11hT and TBP-1 silenced clones were grown in Dulbecco's Modified Eagle Medium (DMEM) supplemented with 10% Fetal Bovine serum and 1 mg/ml puromycin (to maintain selection for h-TERT). U2OS cells were grown in Dulbecco's Modified Eagle Medium supplemented with 10% Fetal Bovine serum.

To obtain *sh*-TBP-1 pool and control pool, 2×10^6^ T11hT cells were transfected by electroporation by making use of a Microporator MP-100 (Digital Bio Technology) either with 3 µg of pSUPERIOR.shTBP-1 or 3 µg of pSUPERIOR.retro.neo; twenty-four hours following transfection, 1 mg/ml G418 was applied to select cells. After four weeks, resistant cells were collected, expanded and analyzed.

Transfection by Lipofectamine2000 were performed as described [12].

Transfection of the T1 clone was performed by the use of a Microporator MP-100 (Digital Bio Technology) using either 2×10^6^ cells with 2 µg of either pcDNA empty vector or pcDNATBP-1 (rescue of cell proliferation, Figure 2E and F) or 1×10^6^ cells with either pcDNA empty vector or pcDNATBP-1 (0.3 or 0.6 µg) (rescue of Akt activation, Figure 5 E). Cells were then plated in DMEM+10% FBS for 24 hrs at 37°C or DMEM without FBS at 37°C and collected for subsequent analysis.

For transient silencing experiments, the duplex siRNA oligomer designed to target human TBP-1 is described in [12]; the duplex siRNA oligomer targeting human MDM2 has the following sequence: 5′- AAGCCAUUGCUUUUGAAGUUA-3′ and was designed as described in [19]. *si*RNA were all synthesized by MWG Biotech, Germany. Either U2OS, T11hT or T1 cells were transfected by Hyperfect (Quiagen, GmBH, Germany) according to the manufacturer's instructions.

### Cell growth analysis, MTS assay, Flow cytometry analysis, Chemoinvasion assay

For cell growth analysis, T11hT parental cell line, T1, T10C and T10E clones, or T11hT, control pool and *sh*-TBP-1 pool, were plated in 100 mm dishes in presence of 10% FBS at the cell density of 1×10^5^ cells/plate. Cells were cultured for 24, 48 and 72 hrs, collected, and counted in a Burker chamber. For growth in the absence of serum, after 6 hrs from plating, medium was removed and replaced with medium without serum. As above, cells have been grown for 24, 48 and 72 hrs, collected and counted. Each point is the result of triplicate samples.

Cell viability was evaluated using the MTS [3-(4,5-dimethylthiazhol-2-yl)-5-(3-carboxymethoxyphenyl)-2-(4-sulfophenyl)-2H-tetrazolium,inner salt] (Cell Titer 96AQueous assay G358 purchased from Promega) colorimetric assay. Briefly, T11hT parental cell line or cells derived from the T1 clone were plated at different cell densities as indicated in 96 well plates (2.5×10^3^/well, 10^3^/well, 3×10^2^ /well) either in DMEM or in DMEM+10%FBS. After six hrs from plating, 1∶5 MTS solution was added to each well and the cells were incubated for 30′ at 37°C. Plates were read on a Microplate Reader (BIO-TEK Instruments, Model Elx800) at 492 nm. Survival was expressed as the percentage of viable cells in treated samples relative to non-treated control cells. All the experiments were repeated in quintuplicate.

The article "A Regulatory Mechanism Involving TBP-1/Tat-Binding Protein 1 and Akt/PKB in the Control of Cell Proliferation" was retracted in 2019. Reasons: manipulated images; duplicated data; unreliable results or conclusions; concerns about the data.

For flow cytometry analysis, T11hT and T1 cells were counted and seeded at 2×10^5^cells/35 mm plate. At 24 hours after plating the medium was replaced and the cells treated with DMEM containing 10% Fetal bovin serum or DMEM without serum. At the indicated time points, cells were collected, centrifuged, washed twice with PBS 1× and then fixed with ice-cold 70% ethanol. Fixed cells were incubated with staining buffer solution (50 µg/ml PI and 50 µg/ml RNase A in PBS pH 7.4) for 20 minute at room temperature in a dark box. Stained cells were analysed in a fluorescence-activated cytometer (DakoCytomation). Data on DNA cell-content were acquired on 20,000 events at a rate of 150±50 events/second and the percentages of cells in the SubG1, G0–G1, S and G2–M phases were quantified with Summit v4.1 software.

Chemoinvasion assays were performed in Boyden chambers using 8 µm pore size PVPF polycarbonate filters coated with 50 µg/ml of Matrigel. 1×105 cells were plated in the upper chamber in serum-free medium. 100 ng/ml EGF or serum free medium was added in the lower chamber. Cells were allowed to migrate for 4 h at 37°C, 5% CO2. To examine basal migration, serum free medium was added to both upper and lower chamber, and migration was allowed for 12 h at 37°C, 5% CO2, in the absence of chemoattractants.

The cells on the lower surface of the filter were then fixed in ethanol, stained with hematoxylin, and counted at 200× magnification (10 random fields/filter).

### Western Blotting, Immunoprecipitations, Insulin treatments, MG132 treatment

Western Blots were performed as described [12]. Antibodies to Akt (used in 1∶1000 dilution), Phospho-Akt Ser473 (used in 1∶1000 dilution), Phospho-GSK-3β/pSer21/9 (used in 1∶1000 dilution), Caspase-3 (1∶1000) and PARP-1 (1∶1000) were purchased from Cell Signalling Technologies, Boston, MA, USA. Antibodies to MDM2 (used in 1∶500 dilution) was purchased from Calbiochem, to Rpt-1 (PSMC2) (used in 1∶6000 dilution), Rpt6 (PSMC5) (used in 1∶6000 dilution) and C8 (used in 1∶6000 dilution) were purchased from BioMol. Anti-Xpress antibody (used in 1∶1000 dilution) was purchased from Invitrogen. Secondary antibodies for Western Blot analysis (goat anti-rabbit IgG-HRP 1∶3000 dilution) were purchased from Santa Cruz Biotechnology, CA, USA. Proteins were visualized with an enhanced chemiluminescence detection system (Amersham ECL ™) and images were taken with ChemiDoc XRS System (Bio-Rad Laboratories) and analysed with the QuantityONE software.

The article "A Regulatory Mechanism Involving TBP-1/Tat-Binding Protein 1 and Akt/PKB in the Control of Cell Proliferation" was retracted in 2019. Reasons: manipulated images; duplicated data; unreliable results or conclusions; concerns about the data.

For insulin treatment, U2OS cells were transfected by Lipofectamine with 0.2 and 0.5 µg of the pcDNATBP-1 plasmid. At 24 hrs after transfection, cells were starved for 4 hrs and then treated with 10 ng/ml insulin for 10′.

To analyze TBP-1 levels following insulin treatments, either U2OS cells or T11hT cells were starved for 4 hrs and then treated with 10 ng/ml insulin for the times indicated.

For immunoprecipitation in U2OS cells, 1.0×10^6^ cells were seeded in 100 mm dishes and transfected with the plasmids indicated in the figure legend. Cells were harvested 24 hours after transfection and cell lysates were prepared as described [12]:

800 µg of whole cell extract were incubated overnight at 4°C with anti-TBP1 (BioMol) or anti-MDM2 C18 (Santa Cruz). Controls of immunoprecipitations were perceived with mouse anti-GFP (Roche) or rabbit anti-Flag (Sigma). Immunocomplexes were collected by incubation with 30 µl of protein A-agarose (Roche Applied Science) at 4°C for 4 hrs. The beads were washed with Co-Ip buffer (50 mM tris-HCL pH 7.5; 150 mM NaCl; 5 mM EDTA; 0,5% Np40), resuspended in 2× loading buffer (Sigma) and loaded on a SDS-8% polyacrylamide gel.

Treatment with proteasome inhibitor was performed as follows: U2OS cells were treated either with DMSO or 10 µM MG132 for five hours. Cells were harvested and total extracts prepared for subsequent analysis as described.

### Constructs

pSUPERIORshTBP-1 has been obtained from pSUPERIOR.retro.neo (Oligoengine) by cloning into BglII-HindII sites a duplex oligonucleotide obtained by MWG-Biotech that could give rise to a short hairpin RNA specifically designed to silence TBP-1 expression.

Oligoseq: ^5′^GATCCCCAACAAGACCCTGCCGTACCTTCAAGAGAGGTACGGCAGGGTCTTGTTTTTTTA^3′^

pCA-Akt plasmid was kindly provided by Prof. G. Condorelli. The MDM2_1–441_ and MDM2_Δ150–230_ expression plasmids were previously described [19].

Plasmids MDM2_S166A_ and MDM2_S166A/S186A_ mutant were generated by Quick Change Site Direct Mutagenesis Kit (Stratagene, La Jolla, CA, USA) and amplified using the following primers:

S166A (F) ^5′^GGAGAGCAATTGCTGAGACAGAAG ^3′^ ,

S166A (R) ^5′^CTTCTGTCTCAGCAATTGCTCTCC ^3′^

S166A/S186A (F) ^5′^ CGCCACAAAGCTGATAGTATTTCCC ^3′^

S166A/S186A (R) ^5′^GGGAAATACTATCAGCTTTGTGGCG^3′^

PCR was performed with a 2720 Thermo Cycler Applied Biosystem.
